This article has been retracted.

# Jordanian Patients' Family Members Need Perceptions in the Critical Care Settings: Nurses' Perspectives versus Family Members' Perspectives in the Context of Health Informatics

**DOI:** 10.1155/2021/4071523

**Published:** 2021-11-27

**Authors:** Hekmat Al-Akash, Roqia Maabreh, Mohannad AbuRuz, Khaled Khader, Abedalmajeed Shajrawi

**Affiliations:** ^1^Faculty of Nursing, Applied Science Private University, Amman, Jordan; ^2^Paramedic Department, Prince Al Hussein Bin Abdulla II Academy for Civil Protection, Amman, Jordan; ^3^Department of Nursing, College of Health Sciences University of Sharjah, Sharjah, UAE; ^4^Faculty of Nursing, Taif University, Taif, Saudi Arabia

## Abstract

**Background:**

An unexpected hospitalization in any of the Critical Care Units (CCUs) is a stressful condition, not only for patients but also for other family members. Research in this field in Jordan is not available. The main objective of this study was to identify the most important needs as perceived by these family members in the light of this stressful event and compare them with the nurses' perceptions of the importance of these needs and also to determine the perception of the needs' importance with the sociodemographic characteristics of both family members and caring nurses.

**Methods:**

This was a cross-sectional study conducted in the period between February and August 2020 among adult family members of patients admitted to the CCUs in hospitals of Jordan from all sectors (public, private, and teaching). The “Critical Care Family Needs Inventory (CCFNI)” questionnaire was administered to 82 family members and 99 CCU nurses to determine the importance of the needs on the inventory. The data were analyzed using descriptive statistics.

**Results:**

The most important need identified by the family members was relevant to the need for proximity (3.64 ± 0.45), followed by information (3.57 ± 0.58), assurance (3.44 ± 0.43), support (3.31 ± 0.62), and comfort (3.21 ± 0.56). Nurses identified the needs for assurance as the highest, followed by information, comfort, and support, whereas proximity was the least need perceived as very important. The top 10 important needs for both family members and nurses were identified. Family members and nurses were only common in 2 of the need statements on the scale. There was no significant association between the sociodemographic characteristics of the sample and the perception of the needs' importance (*p*=0.05).

**Conclusion:**

This study has shown that nurses and family members of patients admitted to CCUs have different perspectives relevant to needs' importance. This should warn nurses to set the needs viewed by family members as a priority. *Implications*. In the CCU settings, in the context of advancing health informatics, families of patients in the ICUs have different needs other than those viewed by nurses. Their needs must be identified and considered.

## 1. Introduction

Family is the basic social system that has been recognized to be a significant source of social and psychological support for its members. This support can help family members maintain their emotional and psychological well-being that ensures the family system's integrity. Any encountered change or disorder by any of those members will lead to disruption in the family system process [1–3]. One of these changes that can negatively affect the family system is the acute illness of any of its members and hospitalization in the Critical Care Units (CCUs). Hospitalization of critically ill patients in any of CCUs often occurs abruptly without any previous warning. It has been proven to be a stressful event not only for the patient but also for other family members [4, 5]. Stress and anxiety experienced by patients' family members are mentioned to be greater than that experienced by the patients themselves during their hospitalization period in the CCUs (Platt, 2016). Increased level of CCU patients' family stress may negatively impact their psychological well-being [6] that may adversely impact the patient's psychological and physiological health status [7].

In response to this difficult situation, the family around the patient may have specific and unique needs [8, 9]. Proper identification of these needs and trying to fulfill them can improve the family members' ability to support their patients. This support can facilitate patients' recovery during CCUs hospitalization [10] and relieve their stress [11], and consequently, patients' stress will be relieved as well. Moreover, meeting the needs of CCU patients' families can improve the healing process [7] and decrease patients' length of stay in CCUs [12, 13].

Molter [14] pioneered the work of family needs in the CCUs. She developed the Critical Care Family Needs Inventory (CCFNI), which was then revised by Leske [15]. It is the most widely used assessment tool for family needs in CCUs. The CCFNI involved the following need categories: information, assurance, support, closeness or proximity, and comfort. Investigating the literature revealed the variable ranking of these needs' importance on the scale. In a review of previous thirty studies conducted between 2000 and 2010, it has been revealed that family members ordered the most important needs as the need for assurance and the need for information [16], where those needs were perceived as being unmet [17, 18]. Unmet family needs may negatively influence patients' family satisfaction and their mental health [19]. Families of patients often view nurses as the most important source to meet their needs [17, 20]. Because nurses are in continuous and close interaction with patients and their families in CCU, they are in an ideal and central position to help family members cope with patient's critical illness in an adaptive way [16]. Nurses may have different perspectives and perceptions regarding the importance of needs other than those of family members. This may represent the reason behind not considering the fulfillment of family needs in the CCU by nurses.

There is limited research describing families and nurses' experiences in CCUs. What is viewed by patient's family members as important might be underestimated by nurses. There are no previous studies that compared the needs' priority perceptions by family members of patients and nurses in the CCUs. Therefore, the main purpose of this study is to clarify the needs' perceptions by family members and compare them with nurses' perceptions of these needs and also to update available knowledge in this regard in Jordan.

## 2. Methods

### 2.1. Design

A nonexperimental, descriptive correlational study design was used for this study.

### 2.2. Settings

Hospitals of different healthcare sectors, public (Royal Medical Services and Ministry of Health Hospitals); private sector; and teaching hospitals' sector, were included in the study.

### 2.3. Sample and Sampling

One hundred family members/visitors of adult patients hospitalized in any of the Critical Care Units and 100 nurses from the same units in the aforementioned hospitals were recruited to participate in this study. Family members were interviewed face-to-face during their availability in the waiting rooms. Nurses were interviewed in the CCUs during their shift hours.

### 2.4. Measurement

A modified Arabic version of the CCFNI was used in this study. The CCFNI was originally developed in English. Both the original CCFNI and the modified Arabic version have 45 Likert-type questions that fall under five dimensions: information (the need for information about the patient in the CCU), proximity (the need for closeness with the patient), assurance (the need for hope regarding patient condition), comfort (the need for facilitation and easiness), and support (including resources and support services). Also, both Arabic and English versions of the CCFNI are a 4-point Likert scale indicating the degree of importance of the given need item statement, where “1” indicates the need statement as “not important at all” to “4” rates the need statement as “very important.” The Arabic CCFNI was reported to be valid and reliable in several studies [18, 21–23].

### 2.5. Ethical Issues

Prior to conducting the study, permission and approval were obtained from the Institutional Review Board (IRB) at the Applied Science Private University as well as the IRB from the selected hospitals where data was gathered. An invitation letter and information sheet were provided to participants. Additionally, informed consent to gain the participants' approval to participate in the study was ensured. Participants were assured that this study would be anonymous; no identifiers of the information about the settings or participants would be disclosed. Also, data will be stored in a locked cabinet, entered data will be in a password-locked PC, and only the researchers will have access to this information. No potential risks or benefits were expected from participation in this study.

## 3. Results

### 3.1. Sample Description

Out of the total recruited sample, 82 CCU patients' family members completed the administered questionnaire. Slightly more than half (51%, *n* = 42) of family members were females. More than two-thirds of the sample aged 20–39 years with a mean of 32.4 ± 9.4; 53 (64.6%) of the patients were males, nearly half of them aged over 60 years with a mean of 52.6 ± 25.8. There were 36 (43.9%) respondents having one of their parents in the CCU; slightly more than half of them spent 5 days or less in the CCU area with a mean of 7.3 ± 8.3 days (Table 1).

Another sample of 99 nurses working in CCU completed the questionnaire. More than half of the nurses aged 30–39 years with a mean of 31.8 ± 4.7 years. Most of them were females (61.6%, *n* = 61) with BSc. degree (79.4%, *n* = 77). Nearly two-thirds of the nurses had 5 years or less of work experience in CCU with a mean of 4.9 ± 3.8, 28.9% (*n* = 28) of them had a CCU training course, and only 4.1% (*n* = 4) of them had a master or Ph.D. degree in CCU (Table 1).

To estimate the mean of the needs' importance perception of both patients' family members and nurses, means ± SDs were calculated. Patients' family members ranked the need for proximity as the highest (mean = 3.64 ± 0.45), followed by information (mean = 3.57 ± 0.58), assurance (3.44 ± 0.43), support (mean = 3.31 ± 0.62), and comfort (3.21 ± 0.56). Nurses identified the needs for assurance as the highest (mean = 3.43 ± 0.32), followed by information (mean = 3.41 ± 0.34), comfort (mean = 3.36 ± 0.33), and support (mean = 3.34 ± 0.36), while proximity (mean = 3.31 ± 0.39) was the least need perceived as very important to nurses (Table 2).

The top 10 most important needs as perceived by CCU nurses are ranked as follows: to “feel that the hospital personnel care about their patient,” “to receive information at least once daily,” “to receive explanations in terms that are understood,” “to have questions answered honestly,” “to know the progress/prognosis,” “to know the exact person as a source for the information,“ “to know accurately what is being done for the patient,” “to be sure the best care possible is being granted to the patient,” “to feel that there is hope,” and “to have their phone calls answered.” Their means  ± SDs are 3.59 ± 0.61; 3.53 ± 0.64; 3.53 ± 0.70; 3.52 ± 0.56; 3.39 ± 0.68; 3.28 ± 0.76; 3.27 ± 0.80; 3.22 ± 0.79; 3.21 ± 0.80; and 3.20 ± 0.68, respectively (Table 3). Their means ± SDs are 3.59 ± 0.61, 3.53 ± 0.64, 5.53 ± 0.70, 3.52 ± 0.56, 3.39 ± 0.68, 3.28 ± 0.76, 3.27 ± 0.80, 3.22 ± 0.79, and 3.22 ± 0.86, respectively (Table 3).

As shown in Table 3, the most important 10 needs as perceived by the family member were ranked as follows: to have flexible visitation hours followed by to stay beside the patient, then to feel that the hospital personnel care about their patient, to receive explanations in terms that are understood to know the progress on the patient, to receive daily information on the patient, to be assured the best care possible is being granted to the patient, to share the care of the patient, to have an area for practicing religious rituals, and to know accurately what is being done for the patient. Their means ± SDs are 3.82 ± 0.39, 3.74 ± 0.49; 3.73 ± 0.57; 3.70 ± 0.54; 3.67 ± 0.55; 3.59 ± 0.63; 3.52 ± 0.63; 3.52 ± 0.65; 3.50 ± 0.62; 3.44 ± 0.67, respectively.

Correlation coefficients between the general mean of all items and sociodemographic variables of patients' family members ranged from 0.027 to 0.406. The highest correlation coefficient (*r* = 0.406) was between “the relation to patient” and the need's priority perceptions. While the weakest correlation was between family member gender and overall mean of all items with only 0.027 (but 0.144 when using Cramer's V). In contrast to others, both age and time variables have a negative correlation coefficient. All values of correlation are nonsignificant (*p* > 0.05) (Tables 4 and 5).

Tables 4 and 5 also clarify the correlation coefficients of the needs' importance perceptions according to the nurses' sociodemographic characteristics. Coefficients ranged from 0.103 to 0.262. The highest correlation coefficient is between nurses' gender and general mean with 0.262, while the lowest is between education and general mean with 0.103 (Cramer's V = 0.117 in case of using binned mean). Although *p*-value for gender is 0.079, which is close to 0.05, still all values of correlation are not significant (*p* > 0.05) with a negative value for age.

## 4. Discussion

Hospitalization in the CCUs has a great impact on patients' physical and psychological integrity, which will impact patients' family coping abilities and perception about the situation of their patients [24]. Nurses are in a central position that hold the responsibility of identifying and fulfilling the needs of their patients' families. This aspect of patient care is a key element of providing holistic healthcare to CCU patients. If family members' immediate needs were identified and fulfilled, desirable consequences for both family members and patients could be achieved; in order to meet family member's needs, CCU nurses must be able to identify these needs accurately.

The current study was conducted to determine the needs' importance in the CCUs that were described by the CCFNI, as perceived by patients' family members compared to nurses. Previous researches conducted in Jordan investigated CCU patients' family needs and highlighted the deficit of care relevant to families. For instance, a previous study in Jordan showed that nurses are not considering the patients' families as part of the holistic approach for patient care [22]. Another previous study in Jordan by Almagharbeh and Alhassan [21] showed that critically ill patients' families need more attention to their psychological needs and involve these needs in their plan of care. The nursing care in CCU in Jordan was almost directed to the management of patient physical status deterioration (focusing on signs and symptoms), ignoring psychological care, with limited attention also to the psychological impact of patients' families during these stressful moments.

It was evident in the results of this study that family members perceived certain needs as very important, whereas nurses did not perceive those needs as the same level of importance. This study attempted to rank the top 10 most important needs from the perspectives of both family members and nurses. Family members and nurses were only common in 2 items with different values of importance perception levels. However, nurses gave a lower perception of importance even for the two common need statements. Similar conclusions were reported in the literature. In one of the available studies, Maxwell and Stuenkel [25] used a 30-item version of Molter and Leske's CCFNI to compare the perception of the needs' importance to families and nurses. Out of the 30 items on the CCFNI, they found a statistically significant difference for 9 items. Family members in the CCUs perceived all items as being of greater importance than did the nurses.

Most of the recent research identified items relevant to assurance as most important to family members [18, 21, 23, 26]. Another recent survey study showed that the most important need identified by the family members in CCUs was the need for assurance, followed by information, proximity, comfort, and support. Moreover, a previous study in Jordan by Almagharbeh and Alhassan [21] revealed that critically ill patients' families perceived assurance, information, and proximity higher than comfort and support needs. Also, patients' family members who had an unconscious/semiconscious relative in the CCUs assigned a higher level of importance to information need compared with those with a conscious relative [27]. These findings are variable and changeable in their priority over time.

The current study came inconsistent with the previous ones as related to the needs' priority perceptions. It showed that the two needs of highest importance were relevant to proximity, which was to have flexible visitation hours and to stay beside the patient. The influence of cultural values held by the family members can be the reason behind this result. In Jordan as an Arabic country, the families used to be larger, extended, and of tighter connectedness with each other. Visiting the patient frequently at the hospital is one of the prominent norms. Family and first-degree relatives or significant others often feel that they do not have to leave the patient; they have to stay around; if something happens, they like to know the new changes immediately at their time of occurrence. At the same time, the healthcare culture and principles relevant to the CCUs do not allow for the presence of patients' families for prolonged periods of time. These units are generally designed on a close basis that imposes separation of the patient from his family. In the Jordanian hospitals in particular, visiting hours often start at the end at a specific time with a slightly wider range during weekends and holidays. The reason behind this policy is to provide a calm environment for the patients and for the healthcare providers, including nurses, doctors, and others to be able to do their jobs toward the patients. Recommendations must be made to have an exception for visitors in the CCU in an organized and noninterrupted manner to ensure the connectedness of patients with their families. Or, the structure of these units can be designated in a way to allow the visitors to see the patients from outside without entering the units. This can mitigate the uncertainty of the families and relieve the stress of both the patients and their families [7]. One of the large medical centers in Jordan started before many years to have a special entrance to the CCU connected to a separate waiting area, with longer visitation hours and assigned a nurse who took the responsibility of organizing the visitation process and answers the questions of the visitors in an attempt to minimize crowds during the visiting hours and allow for connectedness with the patient. Incorporating a balance between families' need to visit and the nurse's need to safely manage the care of their critically ill patient individual has been recommended in the literature [28]. Further studies are indicated to clarify that. Families in this study prioritized the need for proximity over the need for assurance or information. A possible explanation is that the diffusion of information about illnesses is nowadays accessible with only “one click.” People can search and read about diseases using the available or by hand technology. The advancing technology in this regard could influence the families' perceptions that information or assurance is of less importance than proximity. In the past, people relied on doctors and other healthcare professionals as the main source of medical information. Nowadays, with the advancing technology and widespread health informatics and social platforms, people can exchange and find personalized and nonpersonalized health-related information on these platforms [29, 30]. This kind of dissemination of information on social media networks could make people less concerned about seeking information from healthcare professionals [31].

In the past, people tended to ask friends and family for information and advice on how to deal with illness; now, netizens can exchange health information on a large number of virtual communities on social platforms [4]. This kind of digital health community not only helps people find more timely and personalized health-related information [5] but also helps patients discuss and share their medical experience to realize the exchange of personal health information on the platform [6]. Lin et al. [7] built an analysis model based on the data of users' health information exchange experience on Facebook and found that users' interaction behaviors can promote effective health information exchange; however, this kind of interaction behavior is significantly affected by health conditions. In other words, netizens are more inclined to share their health information when they are healthy [8]. Further studies are indicated to confirm that.

Culture shaped the perception of the needs' importance in the current study. A special place to practice religious rituals was among the top ten needs. In Jordan, most of the population is Muslim. They believe in the role of prayers for patient healing and recovery. Females often pray in a private place that is hidden and should not be exposed to strangers. This aspect of supportive care is often ignored while designing the structure of the CCUs. Moreover, Muslim families rely on prayers to alleviate their stress and worries about their patients. Although its often rated as one of the least important needs in a systematic review of literature [32], the role of culture has been emphasized in determining the importance of certain needs [17].

Nurses differ from family members in their perception of the needs' importance. This might be the reason behind not considering the needs of families. In her study, Omari (2009) indicated that none of the 10 most important identified by adult Jordanian family members were perceived as being met. A prior study investigated the perception of CCU nurses on needs of family members of patients admitted to CCU; the CCU nurses classified the family needs for assurance as most important needs, followed by needs for information, need for comfort, needs for closeness, and needs for support [33]. In this study, nurses did not prioritize needs as the family members did. Family members identified their involvement in patient care and have a special place for praying and practicing religious rituals as this is very important, while those needs were identified by nurses as the least important. Involvement of families in their patient member care can create further support for the patient and can help the family feel that they are doing something for their patient. This discrepancy in the perception can lead to an underestimation of the families' emotional needs [34]. Incongruent perception of needs by nurses and families can be a source of conflict among nurses and families, families' dissatisfaction with patient care, and a source of an increased level of stress and anxiety. Consequently, the family might not be able to support their patients during these critical moments. Recommendation has been made in this regard as future interventions, and family involvement decision is to be at different levels of different kinds based on family choice, readiness, and preparedness for that [35].

Regarding the demographic data of patients and their families, the data showed that most patients aged 60 years or more, while the family members were young adults, sons, or daughters. Being a first-degree relative may maximize the perception of the needs' importance, especially the need for proximity as having a flexible visitation and staying at the patient side longer times. In addition, close family members will be more curious to know information. Those family members were too close to the patients and had great concerns with their patients, which reflected on their needs for information and assurance. According to previous literature, most families need adequate information about the current condition of their patients, medical management, and track of disease and prognosis [22, 26, 36]. Unmet informational and assurance needs were found to have an impact on patient's family satisfaction and mental health [19]. Scott, Thomson [19] recommended the provision of oral in addition to structured and written information. This has shown some effect in reducing families' psychological burden and improving their satisfaction with care. Nurses, as a part of the interdisciplinary team and due to long contacts hours with patients and their families, have the core role of providing information to satisfy the most important families' need of awareness about the current and ongoing status of their patients.

Moreover, the need for information is extremely important for all family members irrespective of age, gender, socioeconomic status, and educational level [37]. The family members of the patients hospitalized in the CCU often hope that their questions will be answered clearly and honestly. They also wish to be updated about the new changes in the health status of their patients on the spot [38]. Nurses sometimes tend to give general and unclear information about the patient's condition to alleviate families' anxiety [39]. Studies have declared that informational support from the nurses to the family members of the patient will help them better adapt to stressful conditions and decrease their level of anxiety [40]. Kloos and Daly [41] also emphasized that lack of information and uncertainty about patients' clinical condition is a major factor in increasing family members' depression and anxiety.

The study revealed that the correlation between the mean of all items and sociodemographic variables of patients' family members was not significant (>0.05). Also, a correlation between the mean of all items and sociodemographic variables of nurses was not significant (>0.05). The overall means of all needs as reported by patients' family members and nurses were high (3.10 and 3.0, resp.). The two scores were closed to each other, however, with a different rating of certain needs. This emphasizes the fact that families of patients in the CCU have certain needs that were recognized by nurses and should be fulfilled.

## 5. Conclusion

The study contributes to nursing knowledge about determining the most important needs of patients' families of critically ill patients and nurses. This will help managers understand nurses' needs and develop strategies or prepare an educational program to increase awareness of patients' family needs. But the limitations of the study should be considered regarding the small sample size and the differences in some results of this study and those conducted on non-Arab patients' families.

## Figures and Tables

**Table 1:** Patients, their family members, and nurses' sociodemographic characteristics.

Variable	*N*	%	Variable	*n*	%
Family members' age (years)			Patients' gender		
≤19	4	4.9	Male	53	64.6
20–29	29	35.4	Female	29	35.4
30–39	31	37.8	Relation between patient and family member		
40–49	12	14.6	Son or daughter	36	43.9
50–59	5	6.1	Brother or sister	16	19.5
60+	1	1.2	Parents	10	12.2
Patient's age (years)			Grandson or granddaughter	5	6.1
≤19	12	14.6	Nephew or niece	4	4.9
20–29	2	2.4	Uncle or aunt	3	3.7
30–39	8	9.8	Cousin	2	2.4
40–49	4	4.9	Wife	2	2.4
50–59	18	22	Others	4	4.9
60+	38	46.3	Days of staying in CCU (*n* = 79)		
Family member gender			5 days or less	42	53.2
Male	40	48.8	6–10 days	25	31.6
Female	42	51.2	11–15 days	5	6.3
Total	82	100	16–20 days	4	5.1
			More than 20 days	3	3.8
Nurses SDs:					
Variable	*N*	%			
Age (years)					
20–29	38	38.4			
30–39	56	56.6			
40–49	4	4.0			
50–59	1	1.0			
Gender					
Male	38	38.4			
Female	61	61.6			
Education (*n* = 97)					
Diploma	19	19.6			
Bachelor of science	77	79.4			
Master	1	1.0			
Experience in CCU (*n* = 98)					
5 years or less	64	65.3			
6–10 years	27	27.6			
11–15 years	5	5.1			
More than 15 years	2	2.0			
Having a CCU training course (*n* = 97)					
No	69	71.1			
Yes	28	28.9			
Master/Ph.D. degree in IC (*n* = 97)					
No	93	95.9			
Yes	4	4.1			

**Table 2:** CCFNI subscales ranking according to perceptions of patients' family members and nurses (means ± SD).

CCFNI subscale		CCFNI subscale	
Family members		Nurses	
Subscale	Mean ±SD	Subscale	Mean ±SD
Proximity	3.64 ± 0.45	Assurance	3.43 ± 0.32
Information	3.57 ± 0.58	Information	3.41 ± 0.34
Assurance	3.44 ± 0.43	Comfort	3.36 ± 0.33
Support	3.31 ± 0.62	Support	3.34 ± 0.36
Comfort	3.21 ± 0.56	Proximity	3.31 ± 0.39

**Table 3:** Top 10 need statements (rated as very important) as perceived by family members and CCU nurses.

Rank	Item	Mean	SD	Patients' family members	Mean	SD
	Nurses					
1	To feel that the hospital personnel care about the patient	3.59	0.61	To have flexible visitation hours	3.82	0.39
2	To receive information at least once daily	3.53	0.64	To stay beside the patient	3.74	0.49
3	To receive explanations in terms that are understood	3.53	0.70	To feel that the hospital personnel care about the patient	3.73	0.57
4	To have questions answered honestly	3.52	0.56	To receive explanations in terms that are understood	3.70	0.54
5	To know the progress/prognosis	3.39	0.68	To know the progress/prognosis	3.67	0.55
6	To have their phone calls answered	3.20	0.68			
7	To know the exact person as a source for the information	3.28	0.76	To receive daily information on the patient	3.59	0.63
8	To know accurately what is being done for the patient	3.27	0.80	To be assured the best care possible is being granted to the patient	3.52	0.63
9	To be sure the best care possible is being granted to the patient	3.22	0.79	To share the care of the patient	3.52	0.65
10	To feel that there is hope	3.22	0.86	To have an area to pray and for practicing religious rituals	3.50	0.62
				To know accurately what is being done for the patient	3.44	0.67

**Table 4:** Mean of scores for family needs in CCU for patients' family members according to their sociodemographic characteristics.

Variable	Mean	SD
*Gender*		
Male	3.13	0.51
Female	3.15	0.46
*Age*		
≤ 19	3.26	0.53
20–29	3.18	0.49
30–39	3.09	0.50
40–49	3.08	0.45
50–59	3.10	0.41
60+	3.73	-
*Relation to patient*		
Parents	3.00	0.54
Son or daughter	3.12	0.47
Nephew or niece	2.72	0.40
Cousin	2.66	0.13
Brother or sister	3.24	0.41
Uncle or aunt	3.13	0.56
Grandson or granddaughter	3.68	0.36
Wife	3.30	0.55
Others	3.18	0.54
*Time of staying in CCU*		
5 days or less	3.25	0.46
6–10 days	3.01	0.51
11–15 days	2.65	0.49
16–20 days	3.45	0.15
More than 20 days	2.88	0.26

**Table 5:** Correlation between mean of all items on the CCFNI and sociodemographic variables of patients' family members and nurses.

Family members' SDs	*R*	*P*	Nurses' SDs	*R*	*P*
Age	−0.056	0.619	Age	−0.105	0.301
Gender	0.144	0.426	Gender	0.262	0.079
Gender	0.027	Eta	Gender	0.118	Eta
Relation to patient	0.329	0.339	Education	0.117	0.849
Relation to patient	0.406	Eta	Education	0.103	Eta
Time	−0.134	0.239	Experience	0.164	0.107
Disease	0.339	0.399			
Disease	0.275	Eta			

Eta is used to measure the correlation between nominal and continuous variables, while Cramer's V is used for 2 nominal variables and this is when binning scores to low, medium, and high.

## Data Availability

The data are available upon request from the corresponding author.
